# Budesonide-Loaded Hyaluronic Acid Nanoparticles for Targeted Delivery to the Inflamed Intestinal Mucosa in a Rodent Model of Colitis

**DOI:** 10.1155/2022/7776092

**Published:** 2022-09-27

**Authors:** Seyed Yaser Vafaei, Amir Hossein Abdolghaffari, Reza Mahjub, Seyyed Majid Eslami, Motahareh Esmaeili, Mohammad Abdollahi, Fatemeh Atyabi, Rassoul Dinarvand

**Affiliations:** ^1^Nanomedicine Lab, Department of Pharmaceutics, Faculty of Pharmacy, Tehran University of Medical Sciences, Tehran 1417614411, Iran; ^2^Department of Pharmaceutics, School of Pharmacy, Hamadan University of Medical Sciences, Pajoohesh Sq., Shahid Fahmideh St., Hamadan, Iran; ^3^Department of Toxicology & Pharmacology, Faculty of Pharmacy, Tehran Medical Sciences, Islamic Azad University, Tehran, Iran; ^4^Gastrointestinal Pharmacology Interest Group (GPIG), Universal Scientific Education and Research, Iran; ^5^Department of Pharmacology and Toxicology, Faculty of Pharmacy and Pharmaceutical Sciences Research Center, Tehran University of Medical Sciences, 16th AzarSt., Enqelab Sq., Tehran 1417614411, Iran; ^6^Nanotechnology Research Centre, Faculty of Pharmacy, Tehran University of Medical Sciences, 16th Azar St., Enqelab Sq., Tehran 1417614411, Iran

## Abstract

The aim of the present study was to investigate the therapeutic potential of budesonide- (BDS-) loaded hyaluronic acid nanoparticles (HANPs) for treatment of inflammatory bowel disease (IBD) using an acute model of colitis in rats. The therapeutic efficacy of BDS-loaded HANPs in comparison with an aqueous suspension of the drug with the same dose (30 *μ*g/kg) was investigated 48 h following induction of colitis by intrarectal administration of acetic acid 4% in rats. Microscopic and histopathologic examinations were conducted in inflamed colonic tissue. Tissue concentration of tumor necrosis factor (TNF)-*α* was assessed by ELISA assay kit, while the activity of myeloperoxidase (MPO) was measured spectrophotometrically. Results from in vivo evaluations demonstrated that administrations of BDS-HANPs ameliorated the general endoscopic appearance, quite close to the healthy animals with no signs of inflammation and reduced the cellular infiltration, as well as the TNF-*α* level, and the MPO activity. It was found that delivery by BDS-loaded HANPSs alleviated the induced colitis significantly better than the same dose of the free drug. These data further suggest the potential of HANPs as a targeted drug delivery system to the inflamed colon mucosa.

## 1. Introduction

Inflammatory bowel disease (IBD) is a chronic and relapsing inflammatory condition of the intestinal mucosa. In humans, two major forms, ulcerative colitis (UC) and Crohn's disease, are clinically related and can be differentiated on the basis of histologic manifestation. In the case of UC, the innermost mucosa is involved and the gastrointestinal (GI) tract from the rectum up to the terminal part of the colon is affected [1–3].

In most patients, conventional therapy with anti-inflammatory drugs has been extensively used to treat IBD diseases. Glucocorticoids are considered drug of choice in the treatment of moderate to severe UC. However, their administration is followed by several adverse effects and complications such as immunosuppression, osteoporosis, Cushing's syndrome, bone marrow suppression, hypertension, and glaucoma [4, 5].

Budesonide (BDS) is a second-generation glucocorticoid with high topical efficacy due to high affinity for glucocorticoid receptor and low systemic activity as a result of its extensive first pass metabolism [6]. These characteristics make it the first choice for the induction of remission in moderate to severe colitis [7, 8]. However, available formulations deliver the drug to the ileum and ascending colon and only a small proportion of the drug reaches to the in transverse and descending colon. So, due to limited efficacy and inherent adverse effect of the corticosteroids, budesonide cannot be used for maintenance of remission in UC treatment [9, 10].

Various delivery systems for colon-targeted therapy have been developed; however, there are several controversies in clinical efficacy of these systems due to inter-individual variations and pathologic conditions in IBD [11–13]. Therefore, development of novel drug delivery system (DDS) for specific targeted delivery of BDS to the inflamed area has the benefit of enhanced therapeutic efficacy while maintaining a good safety profile [14–16].

Recently, several studies have focused on the development of colloidal drug carrier systems such as micro- or nanoparticles for targeted delivery to the site of inflammation in IBD therapy [17–20]. It has been reported that the residence time in the gastrointestinal tract can be prolonged by reducing the diameter of particulate carrier [21]. Beside the size, surface charge of the carriers can also influence their targeting efficiency. It was proved that, due to over-expression of cationic proteins in the surface and micro-environment of inflamed cells, particles posing negative charges can potentially exhibit a higher accumulation in inflamed regions [22]. Therefore, negatively charged nanoparticles pose preferential accumulation at the site of inflammation and adhere more strongly to inflamed areas [23, 24]. Moreover, the targeting efficiency can be further increased by preparation of drug carriers bearing targeting moieties [25–27]. Carriers modified with targeting moieties can bind and internalize into the immune cells or the inflamed intestinal mucosa using receptor-mediated endocytosis [28].

In our previous study, we have designed self-assembled HA nanoparticles from amphiphilic conjugates of hyaluronic acid which exhibited negative surface charge due to the ionized carboxylic groups of hyaluronic acid in water [29] and therefore could efficiently interact with cationic proteins in the inflamed region. Moreover, the particles exhibited high affinity to CD44 receptors which are over-expressed in the surface of inflamed colonic epithelial cells. Therefore, it is conceivable that the particles can be targeted to the inflamed colonic epithelial cells through both passive- and active-targeting mechanisms [30].

The aim of the present study was to investigate the *in vivo* anti-inflammatory effects of the BDS-loaded HA nanoparticles against acetic acid-induced colitis in rats. The acetic acid solution induced colitis is a popular experimental model that is widely used to investigate the efficacy of drug delivery systems in animal model of UC [31–33]. Rats were treated intra-rectally by BDS-loaded HA nanoparticles and free BDS suspension. The efficacy of each formulation to improve the lesions was evaluated macroscopically and microscopically. Furthermore, the levels of inflammatory biomarkers including TNF-*α* and myeloperoxidase (MPO) activity were determined in the separated colonic samples.

## 2. Material and Methods

### 2.1. Chemicals

Injectable preparations of phenobarbital sodium were provided from Exir Pharmaceutical Co (Iran). Glacial acetic acid, ethanol (99.9%), diethyl-ether, ethylenediaminetetraacetic acid (EDTA), H_2_O_2_, potassium dihydrogen phosphate (KH_2_PO_4_), di-potasium hydrogen phosphate (K_2_HPO_4_), and sodium chloride were all purchased from Merck™ (Darmstadt, Germany). BDS as the active pharmaceutical ingredient was supplied from Farmabios (Pavia, Italy). Normal saline solution (NaCl 0.9% w/v) was prepared in-house. Formaldehyde was obtained from Mojalali Company (Tehran, Iran). Hexadecyltrimethyl ammonium bromide (HETAB) and O-dianisidine dihydrochloride were purchased from Sigma-Aldrich® (United States). The rat TNF-*α* ELISA kit was supplied from Bender MedSystem™ (Vienna, Austria). In this study, doubled-distilled water which was previously filtered through membrane filters (0.45 *μ*m) was used in all cases. Self-assembled hyaluronic acid nanoparticles containing BDS were prepared, characterized, and reported previously by the authors [30]. All other reagents were of pharmaceutical or analytical grade and were used as received.

### 2.2. Preparation of BDS-Loaded HA Nanoparticles

Amphiphilic hyaluronic acid conjugates were synthesized according to the method reported previously [30]. BDS-loaded HA nanoparticles were prepared according to thin film hydration method. The methodology in brief is as follows: budesonide (5 mg) was dissolved in 5 mL of methanol. The solution was evaporated by a rotary evaporator (50 rpm, 40°C, and 15 min). Afterward, the dried thin films were hydrated by PBS containing HA–DA conjugate powder (10 mg) and stirred overnight at room temperature. The solution was then centrifuged at 10,000 rpm for 10 min, lyophilized, and stored at 4°C for further investigations.

### 2.3. Characterization of BDS-Loaded HA Nanoparticles

#### 2.3.1. Particle Size and Zeta Potential

The size and zeta potential of the nanoparticles was determined using Malvern Zetasizer Nano ZS (Malvern Instruments Ltd., Worcestershire, UK). Samples were diluted in ultra-pure water and measured at 25°C with a scattering angle of 90°.

#### 2.3.2. Drug Content and Encapsulation Efficiency (%EE)

The drug content within BDS-loaded HA nanoparticles was calculated by dissolving the lyophilized powder of drug-loaded nanoparticles (20 mg) in a solvent mixture of methanol/water (1 : 1 v/v) and centrifuged at 10,000 rpm for10 min. The amount of BDS in the supernatant was analyzed by UV/Vis scanning spectrophotometer (Cecil-CE7000-series, Aquarius, UK) at a wavelength of 250 nm. UnloadedHA nanoparticles were used as a blank. The EE% was calculated as the difference between total and free concentrations of BDS, determined in the nanoparticles and ultra-filtrate, respectively.

(1) $$\begin{array}{c} \%\text{EE}=\frac{\text{Total drug content}-\text{Free drug}}{\text{Total drug content}}\times 100,\\ \%\text{Drug content}=\frac{\text{Total drug content}-\text{Free drug}}{\text{Nanoparticles weight}}\times 100. \end{array}$$

#### 2.3.3. Morphological Study

The morphology of the BDS-loaded HA nanoparticles was analyzed by scanning electron microscopy (SEM) and transmission electron microscopy (TEM). For SEM analysis, the dried NPs were coated with gold using gold sputter in a high vacuum evaporator, and the images were observed using a Field Emission Scanning Electron Microscope (FE-SEM, S4160, Hitachi, Japan) operated at an accelerating voltage of 30 kV.

TEM was performed using a Zeiss electron microscope (Zeiss EM10C, Carl ZeissAG, Oberkochen, Germany) operated at an accelerating voltage of 80 kV. A 10-fold diluted aqueous droplet of NPs was placed on carbon-coated copper grids with 1% aqueous solution of phosphotungstic acid (PTA) for negative staining and air-dried at room temperature.

### 2.4. Animals

Adult male Wistar albino rats were provided by the animal breeding house of the Faculty of the Pharmacy of Tehran University of Medical Science (TUMS). Twenty-five rats, weighing 180-200 g, were housed under standard conditions of diet with free access to water, temperature (23 ± 2°C), humidity (55 ± 7%), and 12/12 h light/dark cycle (5 rats in each cage). The current animal study was performed according to the “Principles of Laboratory Animal Care” (NIH publication 82-23, revised in 1985 and 1996). The protocol of the study was approved by the institutional ethical committee of TUMS under code number IR.TUMS.VCR.REC.1396.2341. Animals were randomly designated in different treatment groups and all experiments were blindly performed.

### 2.5. Induction of Colitis

The colitis was induced in rats according to previous studies [34–36]. Prior to colitis induction, rats were fasted for 24 hours, while freely accessed to water. Thereafter, animals were anesthetized by intra-peritoneal (I.P) injection of phenobarbital sodium (45 mg/kg) and the colitis was induced by intra-rectal administration of acetic acid (4% v/v, 2 mL, once in day 1) using a poly-ethylene tube (inserted 6 cm into the colon). In sham or normal group, instead of acetic acid 4%, normal saline solution was administered to rats. Rats were kept under supine trendelenburg position to avoid leaching until complete recovery. There was no mortality in animals, either following colitis induction or after samples administration. Since the animal model of acute colitis was induced with acid solution, welfare of animals has been monitored carefully. Following colitis induction, decreased food intake, bloody diarrhea, and dominant weight loss were observed in rats.

### 2.6. Study Design

24 hours after induction of colitis, based on random classification, the animals were divided into the following five groups (5 rats per group)

1. Group I: Sham or normal group
2. Group II: Colitis-induced rats which received intra-rectal blank nanoparticles
3. Group III: Colitis-induced rats which received intra-rectal free budesonide suspension (30 *μ*g/kg)
4. Group IV: Colitis-induced rats which received intra-rectal hyaloronic acid nanoparticles containing 30 *μ*g/kg of budesonide
5. Group V: Colitis-induced rats which considered as negative control and received no treatment

One mL of each formulation was administered by gavage at days 1, 3, and 5; the sham group and the negative control group received normale saline instead of the formulation. The designated treatment was administered intra-rectally using a poly-ethylene tube with 6 cm of length which was previously inserted into the anus. At the end, rats were anesthetized and the distal segment of their colons were separated, washed (three times with normal saline), and kept for later evolutions. Finally, the animals were sacrificed under anesthesia on day 7 and the colons were removed.

### 2.7. Evaluation and Scoring of Colonic Injury and Inflammation

#### 2.7.1. Macroscopic Evaluations

For macroscopic evaluation, the colon samples were precisely weighted and immediately observed for assessment of severity of the inflammation using a previously reported scoring system [34] as follows: normal appearance, 0; localized hyperaemia without ulcer, 1; linear ulcer without any obvious inflammation, 2; localized linear ulcer with inflammation, 3; obvious ulcers in two or more regions with the length of less than 2 cm, 4; and obvious ulcers with the length of more than 2 cm, 5-8, in a manner that the score was increased by one point by each one centimeter increase in length of ulcers.

#### 2.7.2. Microscopic and Histopathologic Assessment

For microscopic examination, the colonic samples were divided into two equal portions by weight [37]. One portion of each sample was fixed with formaldehyde (10% v/v). The samples were then embedded in paraffin, stained with hematoxylin and eosin, and evaluated microscopically, by a histopathologic that was blinded to treatment allocation, using a light microscope for any evidence of inflammation including edema, presence of granular tissues, infiltration of mono- and poly-nuclear cells, necrosis, and destructions in colonic crypt structures [38]. The severity of the injuries was assessed using the following scoring system; no injuries was counted as 0 point, presence of central necrosis and edema as 1 point, obvious swelling and necrosis in colonic villi as 2 points, observed necrosis and obvious infiltration of neutrophils in sub-mocusal regions as 3 points, and evidence of hemoragia accompanying with extensive necrosis and neutrophils infiltration as 4 points [39]. The other portion of each colonic sample was kept for further evaluation of inflammatory biochemical markers.

### 2.8. Determination of Inflammatory Biochemical Markers

#### 2.8.1. Myeloperoxidase Activity

Myeloperoxidase enzyme can be found in nutrophils, monocytes, and macrophages [34]. The activity of the enzyme is considered an index for quantification of infiltration of polymorph-nuclear cells in one tissue as a result of inflammation. The activity of MPO in a tissue suspension containing neutrophils is linearly correlated to the number of neutrophils.

In this study, the activity of MPO was determined according to previous studies [35]. Briefly, colonic samples were dried, re-weighted, and homogenized in an ice bath containing 10 mL of phosphate buffer (KH_2_PO_4_, 50 mM, pH = 7.4). The homogenate mixtures were then ultra-sonicated and centrifuged for 30 min in 3,500 rpm. Then after, the sediments were separated for determination of the MPO activity, while the supernatants were collected in micro-tubes for determination of TNF-*α*. Each sample (either sediment or supernatant) was kept frozen in -80°C for further analysis.

For performing the MPO activity test and in order to complete and abrupt release of the enzyme from nutrophils, 10 mL phosphate buffer (pH = 7.4) containing 0.5% of hexadecyltrimethyl ammonium bromide (HETAB) and EDTA (10 mM) was added to the settled-down sediments. The mixture was centrifuged for 20 min in 12,000 rpm, following ultra-sonication. The supernatant (100 *μ*L) was collected and mixed with 2.9 mL of phosphate buffer (pH = 7.4) containing O-dianisidine dihydrochloride (0.167 mg/mL) and H_2_O_2_ (0.0005%). Finally, the absorbance of established orange-colored complex was determined in 460 nm, spectrophotometrically.

#### 2.8.2. Determination of the Levels of TNF-*α*

The supernatant of primary colonic homogenate was treated by a sandwich type ELISA technique (The Bender Medsystem™ rat TNF-*α* ELISA kit), according to the instruction provided by the manufacturer [40]. Samples were analyzed by an ELISA-reader at wavelengths of 450 nm Vs 650 nm. The total protein concentration was determined using Lowry method protein assay.

### 2.9. Statistical Analysis

Statistical analyses were performed using the Stats-Direct® program (V.3.0.107, Merseyside, United Kingdom). The one-way ANOVA test of multiple comparisons followed by Tukey's post hoc test was applied for data comparisons. All other analyses were performed using Student's *t*-test. Differences were considered statistically significant at ∗*p* < 0.05. The results are expressed as the means ± SD (SD: standard deviation).

## 3. Results

### 3.1. Preparation and Characterization of BDS-Loaded HA Nanoparticles

Amphiphilic hyaluronic acid conjugates with degree of substitution (DS) of 34% were synthesized according to our previous study [30]. Successful conjugation was confirmed by 1H NMR and FTIR spectral analysis. Blank HA nanoparticles with negative charge and diameter of 177 ± 6 were prepared. HA is a biocompatible, negatively charged linear polysaccharide composed of N-acetyl glucosamine and D-glucuronic acid as a repeating unit. The negative charge of HA nanoparticles is attributed to the ionized carboxylic groups of hyaluronic acid in water [29]. BDS was loaded into the hydrophobic core of HA nanoparticles by thin film hydration method. FTIR analysis and DSC confirmed the loading of the drug into the HA nanoparticles. The characteristics of BDS-loaded HA–DA nanoparticles are summarized in Table 1. The amount of BDS present in hydrophobic core of HA–DA nanoparticles was 9.3% and the encapsulation of the drug resulted in an increase in the particle size. The BDS-loaded HA nanoparticles exhibited a diameter of 266 ± 16 nm. Zeta potentials of blank HANPs and BDS-loaded HANPs were − 19.66 ± 0.74 mV and − 3.98 ± 0.46 mV, respectively. By imaging with SEM and TEM (Figure 1), an acceptable spherical morphology was observed.

### 3.2. Macroscopic Evaluations

Figures 2(a) and 2(b) show, respectively, opened colon of control rats that received normal saline 0.9% (v/v) and of rats after induction of colitis with acetic acid, sacrificed on day 7. The group of animals sacrificed 7th day after colonic administration of acetic acid showed necrotic changes and presented extensive ulcers and severe hemoragia. In Figures 2(c)–2(e), opened colons of groups II, III, and IV are presented, respectively. Colons from group II (Figure 2(c)) showed the presence of necrotic zone, edema, and severe hemoragia. Colons from group III (Figure 2(d)) present a little hyperaemia and ulcers; interestingly, in group IV, which were treated by BDS- containing nanoparticles (Figure 2(e)), colons appeared healthy. Scoring data obtained from macroscopic evaluations of separated colons are illustrated in Figure 3. As shown in the figure, the separated samples from colonic segments in sham group had normal appearance (i.e., score 0). However, induction of colitis in group II (received blank nanoparticles) and group V of animals (control group) caused edema, extensive ulcers, and severe hemoragia, exhibiting the highest colonic injury scores among other groups (*p* < 0.001). Although intra-rectal administration of free BDS significantly reduced the inflammation scores in group III of animals compared with control group (*p* < 0.001), nonetheless hyperaemia and ulcers could still be observed in the samples. Interestingly, in group IV, which were treated by BDS-containing nanoparticles, the scores of colonic injuries were the lowest among the other groups (*p* < 0.05), indicating the effectiveness of therapy in reducing the inflammation (Figure 3).

### 3.3. Microscopic Evaluation

Histophathological images of experimental samples are represented in Figures 4(a)–4(e). Histological assessment of sham group (group I) revealed normal epithelial cells with no pathological evidence (Figure 4(a)). In contrast, identical to control group, microscopic images obtained from samples separated from group II (received blank nanoparticles) showed complete degeneration of mucosal epithelium, extensive ulcers, extensive destruction of crypts, extensive inflammation, sub-mucosal infiltration of inflammatory cells, edema, and hemoragia (Figures 4(b) and 4(c)). In group III (treated by free BDS suspension), regeneration of mucosal epithelium had been initiated; however, colitis was not completely revealed (Figure 4(d)). Although the extent of infiltration of inflammatory cells was reduced in sub-mucosal, but some evidence of infiltration was still present. In group IV, degenerated regions including epithelium, crypts, and muscles were mostly regenerated. However, incomplete formation of crypts and epithelial cells and mild inflammation as well as limited infiltration of inflammatory cells to mucosal and sub-mucosal area was still present (Figure 4(e)). Rats in group IV exhibited the lowest injury score among all colitis-induced animals (Figure 5).

### 3.4. Determination MPO Activity

As shown in Figure 6, the MPO activity in the control group was significantly higher than the appropriate value in sham group (*p* < 0.001). Although the enzyme activity was slightly lower in group II, the difference with control group was not significant (*p* > 0.05). On the other hand, administration of intra-rectal free BDS resulted in significantly lower enzyme activity (*p* < 0.001). As expected, the MPO activity in group IV was approximately 1.5-fold lower than animals in which BDS suspension were administered.

### 3.5. Determination of the Levels of TNF-*α*

It is obvious that in control group (i.e., group V), secretion of TNF-*α* was significantly raised by approximately 4-fold in comparison with sham group (*p* < 0.001). Although the levels of the cytokine in group II of animals which received blank nanoparticles were slightly greater than the corresponding values in control group, however statistical analysis revealed no significant differences (*p* > 0.05). Comparing with control group, administration of intra-rectal free BDS caused significant reduction in levels of the inflammatory cytokine (*p* < 0.05), but the lowest level of TNF-*α* was observed in group IV that were treated with BDS-containing nanoparticles (*p* < 0.05) (Figure 7).

## 4. Discussion

In our previous study using cellular model of inflamed intestinal mucosa (CACO-2 cells), we showed that BDS-loaded HANPs demonstrated stronger anti-inflammatory effect on IL-8 and TNF-*α* secretion compared with the same dose of free drug [30]. The aim of this study was to evaluate the therapeutic efficacy of BDS-loaded HANPs using acetic acid-induced colitis in rat model. Acetic acid-induced colitis is one of the most commonly used animal models for evaluation of therapeutic efficacy of drugs for IBD and has similar histological and clinical features to that of human colitis [36]. The therapeutic efficacy of BDS-loaded HANPs was investigated 48 h following colitis induction through macroscopic, histological, and biochemical analysis.

Administrations of BDS-loaded HANPs significantly alleviated acetic acid-induced colitis in comparison with that of control (*p* < 0.05). Administrations of BDS-HANPs ameliorated the general endoscopic appearance quite close to the healthy mice groups with no signs of inflammation and reduced the cellular infiltration and the levels of inflammatory cytokines. On the basis of histological evaluation, treatment with BDS when administered as free drug showed some amelioration of the inflammation, but no complete recovery was observed due to its extensive hepatic metabolism [40–42]. Animals treated with BDS-loaded HANPs exhibited colonic architecture similar to control group, indicating improved therapeutic efficiency and the difference was statistically significant.

Myeloperoxidase (MPO) is the most abundant protein in neutrophils and plays an important role in the initiation and progression of inflammation [34]. In this study, the MPO activity was used as a standard test in animal models and was detected as a parameter for determining the extent and severity of inflammation. Untreated animals suffering from colitis showed a significant higher level of MPO in comparison with healthy rats. Both BDS and BDS-loaded HANPs exhibited significant reduction in MPO activity; however, the efficacy of BDS-loaded HANPs was statistically significant in the study (*p* < 0.05).

In inflamed areas, activation of innate immune cells such as macrophages led to the secretion of pro-inflammatory cytokines such as TNF-*α* [43]. A significant reduction was observed in secretion of TNF-*α* in BDS-loaded HANPs-treated group in comparison with other treated groups, highlighting the contribution of HANPs in healing effect of BDS.

In a cellular model, physicochemical properties of the nanoparticles, including size and charge, significantly affected their passive targeting potential to inflamed intestinal areas, thus avoiding rapid elimination. In this study, similar results were observed (Figure 3(e)). Herein, we confirmed the promising potential of HA nanoparticles as a targeted drug delivery system for IBD treatment.

## 5. Conclusion

In this study, the in vivo efficacy of a colon-targeted delivery system containing BDS was evaluated in acetic acid-induced rat colitis model. In our previous study, BDS-containing self-assembled nanoparticles composed of amphiphilic conjugate of decylamine-hyaluronic acid were prepared and physico-chemically characterized. It was shown that these nanoparticles could target inflamed colonic tissues through specific interactions with CD44 receptors, which were over-expressed in inflamed tissues.

In the current study, it was demonstrated that intra-rectal administration of BDS-HANPs could relieve the macroscopic evidence of inflammation. Although in microscopic evaluation of tissues, complete remission was not found, but it was confirmed that incorporation of BDS into the NPs was effective in regeneration of inflammation-induced degenerated muscles, epithelial cells, and crypts. Moreover, it was demonstrated that the drug delivery system could significantly reduce the MPO activity and the secretion of TNF-*α* in comparison with animals that received free BDS suspension. In conclusion, BDS-HANPs exhibit more efficiency in reduction of colitis compared with free BDS and it can be suggested as an effective, alternative candidate for treatment of IBD.

## Figures and Tables

**Figure 1:** (a) The size distribution (a) and morphologies (b) SEM image. (c) TEM image (bar = 500 nm) of the BDS-loaded HA NPs (b).

**Figure 2:** Photographs of the colon of rat after the induction of colitis with acetic acid sacrificed on day 7: (a) (sham or normal group; group I), (b) (untreated acetic acid group; group V), (c) (blank nanoparticles treated group; group II), (d) (budesonide suspension treated group; group III), (e) (budesonide-loaded HA nanoparticle treated group; group IV).

**Figure 3:** Macroscopic scoring of colonic injuries in different animal groups. ^a^Significantly different from sham (group I) (*p* < 0.05). ^b^Significantly different from control (group V) (*p* < 0.05). ^c^Significantly different from the blank-treated group (group II) (*p* < 0.05),^d^ Significantly different from the BDS Susp-treated group (group III) (*p* < 0.05).

**Figure 4:** Microscopic images of colonic tissues obtained from (a) sham or normal group (group I); (b) control group (group V); (c) animal group which received blank nanoparticles (group II); (d) animal group which received free BDS (group III); (e) animal group which received BDS nanoparticles (group IV).

**Figure 5:** Microscopic scoring of colonic injuries in different animal groups. ^a^Significantly different from sham (group I) (*p* < 0.05). ^b^Significantly different from control (group V) (*p* < 0.05). ^c^Significantly different from the blank-treated group (group II) (*p* < 0.05). ^d^Significantly different from the BDS Susp-treated group (group III) (*p* < 0.05).

**Figure 6:** MPO activity in colonic samples of different animal groups. (a) Significantly different from sham (group I) (*p* < 0.05). (b) Significantly different from control (group V) (*p* < 0.05). (c) Significantly different from the blank-treated group (group II) (*p* < 0.05). (d) Significantly different from the BDS Susp-treated group (group III) (*p* < 0.05).

**Figure 7:** Level of TNF-*α* in colonic sample of different animal groups. (a) Significantly different from sham (group I) (*p* < 0.05). (b) Significantly different from control (group V) (*p* < 0.05). (c) Significantly different from the blank-treated group (group II) (*p* < 0.05). (d) Significantly different from the BDS Susp-treated group (group III) (*p* < 0.05).

**Table 1:** Characterization of budesonide-loaded HA–NPs (*n* = 3; data are expressed as mean ± SD).

NPs characterization					
	Size (nm)	Zeta potential (mV)	PdI	BDS content (Wt. %)^a^	Encapsulation efficiency (%)^b^
Blank HA NPs	177 ± 6	- 19.66 ± 0.74	0.22 ± 0.03	—	—
BDS loaded HANPs	266 ± 16	- 3.98 ± 0.46	0.29 ± 0.08	9.3 ± 0.45	18.6

^a^Calculated by dividing the encapsulated BDS with the predetermined amount of BDS loaded HA–NPs. ^b^Calculated by dividing the encapsulated BDS with initial BDS amount.

## Data Availability

Data are available on request.

## References

[1] Baumgart D. C., Sandborn W. J. (2007). Inflammatory bowel disease: clinical aspects and established and evolving therapies. *The Lancet*.

[2] Khor B., Gardet A., Xavier R. J. (2011). Genetics and pathogenesis of inflammatory bowel disease. *Nature*.

[3] Sartor R. B. (2006). Mechanisms of disease: pathogenesis of Crohn’s disease and ulcerative colitis. *Nature Clinical Practice Gastroenterology & Hepatology*.

[4] Cai Z., Wang S., Li J. (2021). Treatment of inflammatory bowel disease: a comprehensive review. *Frontiers in Medicine*.

[5] Curkovic I., Egbring M., Kullak-Ublick G. A. (2013). Risks of inflammatory bowel disease treatment with glucocorticosteroids and aminosalicylates. *Digestive Diseases*.

[6] Chopra A., Pardi D. S., Loftus E. V. (2006). Budesonide in the treatment of inflammatory bowel disease: the first year of experience in clinical practice. *Inflammatory Bowel Diseases*.

[7] Sherlock M. E., MacDonald J. K., Griffiths A. M., Steinhart A. H., Seow C. H., Cochrane IBD Group (2015). Oral budesonide for induction of remission in ulcerative colitis. *The Cochrane Database of Systematic Reviews*.

[8] Iborra M., Alvarez-Sotomayor D., Nos P. (2014). Long-term safety and efficacy of budesonide in the treatment of ulcerative colitis. *Clinical and Experimental Gastroenterology*.

[9] Edsbäcker S., Bengtsson B., Larsson P. (2003). A pharmacoscintigraphic evaluation of oral budesonide given as controlled-release (Entocort) capsules. *Alimentary Pharmacology & Therapeutics*.

[10] Quetglas E. G., Armuzzi A., Wigge S. (2015). Review article: The pharmacokinetics and pharmacodynamics of drugs used in inflammatory bowel disease treatment. *European Journal of Clinical Pharmacology*.

[11] Carrette O., Favier C., Mizon C. (1995). Bacterial enzymes used for colon-specific drug delivery are decreased in active Crohn’s disease. *Digestive Diseases and Sciences*.

[12] Nugent S. G., Kumar D., Rampton D. S., Evans D. F. (2001). Intestinal luminal pH in inflammatory bowel disease: possible determinants and implications for therapy with aminosalicylates and other drugs. *Gut*.

[13] Fallingborg J., Christensen L. A., Jacobsen B. A., Rasmussen S. N. (1993). Very low intraluminal colonic pH in patients with active ulcerative colitis. *Digestive Diseases and Sciences*.

[14] Yasmin F., Najeeb H., Shaikh S. (2022). Novel drug delivery systems for inflammatory bowel disease. *World Journal of Gastroenterology*.

[15] Antunes J. C., Seabra C. L., Domingues J. M. (2021). Drug targeting of inflammatory bowel diseases by biomolecules. *Nanomaterials*.

[16] Hua S. (2020). Advances in oral drug delivery for regional targeting in the gastrointestinal tract - influence of physiological, pathophysiological and pharmaceutical factors. *Frontiers in Pharmacology*.

[17] Beloqui A., Coco R., Alhouayek M. (2013). Budesonide-loaded nanostructured lipid carriers reduce inflammation in murine DSS-induced colitis. *International Journal of Pharmaceutics*.

[18] Lin M., Dong L., Chen Q. (2021). Lentinan-based oral nanoparticle loaded budesonide with macrophage-targeting ability for treatment of ulcerative colitis. *Frontiers in Bioengineering and Biotechnology*.

[19] Sinhmar G. K., Shah N. N., Chokshi N. V., Khatri H. N., Patel M. M. (2018). Process, optimization, and characterization of budesonide-loaded nanostructured lipid carriers for the treatment of inflammatory bowel disease. *Drug Development and Industrial Pharmacy*.

[20] Ali H., Weigmann B., Neurath M. F., Collnot E. M., Windbergs M., Lehr C. M. (2014). Budesonide loaded nanoparticles with pH-sensitive coating for improved mucosal targeting in mouse models of inflammatory bowel diseases. *Journal of Controlled Release*.

[21] Lamprecht A., Schäfer U., Lehr C.-M. (2001). Size-dependent bioadhesion of micro- and nanoparticulate carriers to the inflamed colonic mucosa. *Pharmaceutical Research*.

[22] Jubeh T. T., Barenholz Y., Rubinstein A. (2004). Differential adhesion of normal and inflamed rat colonic mucosa by charged liposomes. *Pharmaceutical Research*.

[23] Collnot E. M., Ali H., Lehr C. M. (2012). Nano- and microparticulate drug carriers for targeting of the inflamed intestinal mucosa. *Journal of Controlled Release*.

[24] Schmidt C., Lautenschlaeger C., Collnot E. M. (2013). Nano- and microscaled particles for drug targeting to inflamed intestinal mucosa: a first in vivo study in human patients. *Journal of Controlled Release*.

[25] Varshosaz J., Emami J., Ahmadi F. (2011). Preparation of budesonide-dextran conjugates using glutarate spacer as a colon-targeted drug delivery system: in vitro/in vivo evaluation in induced ulcerative colitis. *Journal of Drug Targeting*.

[26] Mladenovska K., Raicki R. S., Janevik E. I. (2007). Colon-specific delivery of 5-aminosalicylic acid from chitosan-Ca-alginate microparticles. *International Journal of Pharmaceutics*.

[27] Lehr C. M. (2000). Lectin-mediated drug delivery:. *Journal of Controlled Release*.

[28] Mura C., Nacher A., Merino V. (2011). *N*-Succinyl-chitosan systems for 5-aminosalicylic acid colon delivery: In vivo study with TNBS-induced colitis model in rats. *International Journal of Pharmaceutics*.

[29] Schanté C. E., Zuber G., Herlin C., Vandamme T. F. (2011). Chemical modifications of hyaluronic acid for the synthesis of derivatives for a broad range of biomedical applications. *Carbohydrate Polymers*.

[30] Vafaei S. Y., Esmaeili M., Amini M., Atyabi F., Ostad S. N., Dinarvand R. (2016). Self assembled hyaluronic acid nanoparticles as a potential carrier for targeting the inflamed intestinal mucosa. *Carbohydrate Polymers*.

[31] Ahmed O., Abdel-Halim M., Farid A., Elamir A. (2022). Taurine loaded chitosan-pectin nanoparticle shows curative effect against acetic acid-induced colitis in rats. *Chemico-Biological Interactions*.

[32] Kassab R. B., Elbaz M., Oyouni A. A. A. (2022). Anticolitic activity of prodigiosin loaded with selenium nanoparticles on acetic acid-induced colitis in rats.

[33] Qelliny M. R., Aly U. F., Elgarhy O. H., Khaled K. A. (2019). Budesonide-loaded Eudragit S 100 nanocapsules for the treatment of acetic acid-induced colitis in animal model. *AAPS PharmSciTech*.

[34] Wallace J. L., Whittle B. J., Boughton-Smith N. K. (1985). Prostaglandin protection of rat colonic mucosa from damage induced by ethanol. *Digestive Diseases and Sciences*.

[35] Can G., Ayvaz S., Can H. (2015). The Syk inhibitor fostamatinib decreases the severity of colonic mucosal damage in a rodent model of colitis. *Journal of Crohn's & Colitis*.

[36] Mizoguchi A. (2012). Animal models of inflammatory bowel disease. *Progress in Molecular Biology and Translational Science*.

[37] Fakhraei N., Abdolghaffari A. H., Delfan B. (2014). Protective effect of hydroalcoholic olive leaf extract on experimental model of colitis in rat: involvement of nitrergic and opioidergic systems. *Phytotherapy Research*.

[38] Neurath M. F., Fuss I., Pasparakis M. (1997). Predominant pathogenic role of tumor necrosis factor in experimental colitis in mice. *European Journal of Immunology*.

[39] Rosenberg L., Nanda K. S., Zenlea T. (2013). Histologic markers of inflammation in patients with ulcerative colitis in clinical remission. *Clinical Gastroenterology and Hepatology*.

[40] Edsbacker S., Andersson P., Lindberg C., Paulson J., Ryrfeldt A., Thalén A. (1987). Liver metabolism of budesonide in rat, mouse, and man. Comparative aspects. *Drug Metabolism and Disposition*.

[41] Greenberg G. R., Feagan B. G., Martin F. (1994). Oral budesonide for active Crohn’s disease. *The New England Journal of Medicine*.

[42] Jönsson G., Aström A., Andersson P. (1995). Budesonide is metabolized by cytochrome P450 3A (CYP3A) enzymes in human liver. *Drug Metabolism and Disposition*.

[43] Begue B., Wajant H., Bambou J. C. (2006). Implication of TNF-related apoptosis-inducing ligand in inflammatory intestinal epithelial lesions. *Gastroenterology*.

